# LONG-TERM OUTCOMES OF LIGATION OF INTERSPHINCTERIC FISTULA TRACT FOR COMPLEX FISTULA-IN-ANO: MODIFIED OPERATIVE PROCEDURE EXPERIENCE

**DOI:** 10.1590/0102-672020180001e1404

**Published:** 2018-12-06

**Authors:** Ke WEN, Yun-Fei GU, Xue-Liang SUN, Xiao-Peng WANG, Shuai YAN, Zong-Qi HE, Shu-Guang ZHEN

**Affiliations:** 1 Nanjing University of Chinese Medicine, Colorectal Surgery, Nanjing, Jiang su, China;; 2 Suzhou Affiliated Hospital of Nanjing University of Chinese Medicine, Colorectal Surgery, Su zhou, Jiang su, China

**Keywords:** Complex fistula-in-ano, Ligation of the intersphincteric fistula tract, Modified operative procedure, Fístula complexa no ano, Ligadura do trato da fístula interesfincteriana, Procedimento operatório modificado

## Abstract

**Background:**

It is important but difficult to treat complex fistula-in-ano due to the high recurrent rate and following incontinence. Ligation of the intersphincteric fistula tract (LIFT), a novel surgical procedure with the advantage of avoiding anal incontinence, has a variable success rate of 57-94.4 %.

**Aim:**

To evaluate the long-term outcomes of modified LIFT operative procedure - ligation of intersphincteric fistula tract - to treat complex fistula-in-ano.

**Methods:**

Retrospective analysis of 62 cases of complex fistula-in-ano. The group was treated with the modified approach of LIFT (curved incision was made in the anal canal skin; purse-string suture was performed around the fistula; the residual fistulas were removed in a tunnel-based way) and had a follow-up time of more than one year. Patient´s preoperative general condition, postoperative efficacy and their anal function were compared.

**Results:**

The median age of the participants was 34, and 43 (69.4%) cases were male. Forty-one (66.1%) cases were of high transsphincteric fistula, four (6.5%) cases of high intrasphincter fistula, and 17 (27.4%) cases of anterior anal fistula in female. The median follow-up duration was 24.5 (range, 12-51) months. The success rate in the end of follow-up was 83.9% (52/62). The anorectal pressure and Cleveland Clinic Florida Fecal Incontinence (CCF-FI) evaluated three months before and after the operation did not find apparent changes.

**Conclusions:**

Compared with LIFT, the modified LIFT remarkably reduces postoperative failure and the recurrence rate of complex fistula with acceptable long-term outcomes.

## RESUMO

**Racional:**

É importante, mas difícil de se tratar fístula anal complexa devido à alta taxa de recorrência e de incontinência pós-operatória. A ligadura do trajeto da fístula interesfincteriana (LIFT) - um novo procedimento cirúrgico com a vantagem de evitar a incontinência anal - tem taxa de sucesso variável entre 57-94,4%.

**Objetivo:**

Avaliar os resultados em longo prazo do procedimento cirúrgico LIFT modificado - ligadura do trato interesfincteriano com fístula - para tratar fístula complexa anal.

**Métodos:**

Análise retrospectiva de 62 casos de fístula complexa no ânus tratados com abordagem modificada de LIFT (incisão curva na pele do canal anal; sutura em bolsa realizada em torno da fístula; as fístulas residuais removidas em um túnel) e teve tempo de acompanhamento de mais de um ano. A condição geral pré-operatória dos pacientes, a eficácia pós-operatória e a função anal foram comparadas.

**Resultados:**

A mediana de idade dos participantes foi de 34 anos, e 43 (69,4%) dos casos eram de homens. Quarenta e um (66,1%) casos eram de fístula transesfincteriana alta, quatro (6,5%) de fístula intra-esfincteriana alta e 17 (27,4%) de fístula anal anterior em mulheres. A mediana da duração do acompanhamento foi de 24,5 meses (12-51). A taxa de sucesso no final do acompanhamento foi de 83,9% (52/62). A pressão anorretal e a Incontinência Fecal da Cleveland Clinic Florida (CCF-FI) avaliadas três meses antes e após a operação não encontraram alterações aparentes.

**Conclusões:**

Comparado com o LIFT, o LIFT modificado reduz notavelmente a falha pós-operatória e a taxa de recorrência de fístula complexa com resultados aceitáveis em longo prazo.

## INTRODUCTION

Complex fistula-in-ano is one of the refractory diseases of anorectal surgery. Classic treatment for it, such as fistulotomy and/or seton placement, is associated with a high recurrence or insufficient protection of anal function^3^. Sphincter-preserving technique, on the other hand, seems to preserve faecal continence at the expense of higher recurrence rate^5^. In 2007, Rojanasakul from Thailand reported a novel surgical sphincter-sparing technique, known as the ligation of intersphicteric fistula tract (LIFT)^14^. Performed via the normal anatomical gap without internal and external sphincter injury, it prevents the decrease of postoperative anal autonomous control. As its cure rate ranges from 57-94.4% according to meta-analysis and retrospective analysis^7^, several studies attempt to improve the procedure so as to further increase the cure rate. However, it turns out that the internal and external sphincter integrity is damaged to some degrees, which strays from the idea of upholding the integrity of sphincter by LIFT surgery. 

Therefore, the present study aims to improve LIFT surgery to further increase its cure rate of complex fistula-in-ano. On the principle of protecting the integrity of the internal and external sphincter, we modify LIFT operative procedure from the following three aspects: curved incision in the anal canal skin; purse-string suture performed around the fistula; residual fistulas removed in a tunnel-based way.

## METHODS

A retrospective review was carried out among 62 patients of complex fistula-in-ano treated with modified LIFT in Suzhou Affiliated Hospital of Nanjing University of Chinese Medicine between January 2013 and December 2016. The study was approved by Ethics Committee Suzhou Affiliated Hospital of Nanjing University of Chinese Medicine (2013 NL-056-02). All the participants were diagnosed with complex fistula-in-ano by using perianal MRI before operation^4^, without significant abnormalities of external and internal sphincter according to anorectal pressure determination.

Inclusion criteria were: 1) patient over 18 years old; 2) with complex cryptoglandular anal fistula with newly-diagnosed fistula-in-ano; 3) no significant abnormalities of external and internal sphincter in anorectal pressure measurement; 4) the patient want to be submitted to LIFT surgery and has signed the informed consent before the operation. 

Exclusion criteria were: 1) the patient refused LIFT surgery and chose other surgical treatment; 2) no Crohn’s disease; 3) another inflammatory bowel disease or malignancy.

The primary end point was success after surgery for anal fistula using the LIFT procedure. Success after the LIFT procedure was defined as complete healing of the surgical intersphincteric wound and the external opening without any sign of recurrence. Failure was defined as a clinical diagnosis of fistula recurrence at any time in the postoperative follow-up defined by clinical interview, physical examination.

### Operative procedure

The patients were placed in the prone jackknife position after successful combined spinal epidural anesthesia. Based on perianal MRI examination before surgery, fistula tracts and internal openings were found with the assistance of hydrogen peroxide solution and probe. At first, the position of intersphincteric groove was confirmed with the examining finger. A1.5-2.0 cm curved incision was made at the anal canal skin (Figure 1) to disconnect the intersphincteric fistula between the internal and external sphincters before it reached the intersphincteric groove; the intersphincteric fistula lifted with right angle forceps. Purse-string suture around the fistula was then introduced for the ligation of the fistula at the side of internal sphincter with 3/0 vicryl close to the lateral side of internal anal sphincter (Figure 2). Afterwards, hydrogen peroxide was injected from the external opening to verify that fistula ligation was completed. Similarly, purse-string suture around the fistula was performed for the ligation of the fistula at the side of external sphincter with 3/0 vicryl close to the interior side of external anal sphincter. Hydrogen peroxide was injected again, after the fistula between the two ligation threads was cut, to verify if fistula ligation near the external sphincter was completed. Next, the residual fistulas were removed in a tunnel-based way to the external sphincter border (Figure 3). The external opening was unclosed for drainage. Intersphincteric was sutured with 4/0 vicryl, perianal skin and the subcutaneous arc-shaped incision were sutured with 3/0 vicryl.

**FIGURE 1:** Curved incision in the anal canal skin

**FIGURE 2:** Purse-string suture around the fistula

**FIGURE 3:** The residual fistulas removed in a tunnel-based way

As for female with high intersphincteric fistulas and anterior intersphincteric anal fistula, the tract was cored out from the external opening. Once it penetrated the internal sphincter, the suture kept close to the outside sphincter and a purse-string suture was to stitch in a circle around the tract to tie it up. The external opening was unclosed for drainage.

After operation, the patients were administrated with soft diet and their voluntary defecation was controlled within 48 h. Controlled diet and medication promised soft and smooth stool of the patients. The conventional intravenous antibiotics were given for 48 h to prevent infection. In addition, sitz bath was forbidden and 0.5% iodophor was used for daily cleaning and dressing after stooling. Vaseline gauze was placed inside the external opening for drainage. Furthermore, outpatient visit was required two weeks after discharge. The follow-up information was collected by specific personnel through questionnaires at outpatient clinic. Finally, Cleveland Clinic Florida Fecal Incontinence (CCF-FI)^8^ was applied to evaluate the autonomous control function of the anal sphincter three months before and after the operation and in the end of the follow-up. The anorectal pressure determination was performed to evaluate anal functions and monitor the anal canal resting pressure and maximum contractive pressure three months before and after the operation respectively. The follow-up ended on December 2017.

### Statistical analysis

Statistic software SPSS22.0 was utilized in the present study. Continuous data were presented as mean (SD) or median (interquartile range), for parametric and nonparametric data. Categorical data were reported as percentage proportion. A Student’s t-test was used to determine the significance of the difference in one group before and after operation, and Chi-square test was used for enumeration data. Differences were considered significant for *p<*0.05.

## RESULTS

The basic information and characteristics of fistula were summarized in Table 1. Consecutive patients with newly diagnosed complex fistula-in-ano were operated on using the modified LIFT technique, 43 patients were male. Median age was 34 (22-63) years. Forty-one patients had high transsphincteric fistula, four high intrasphincter and 17 anterior anal fistula, in female; eight patients had horseshoe fistula, while 18 perianal abscess surgery history. Previous seton drainage was not used in any case. There were seven cases of incision dehiscence and infection occurred after operation. For patients with intersphincteric incision dehiscence, the incision achieved healing by secondary intention through incision dressing and external application of mupirocin ointment. The median follow-up duration was 24.5 (12-51) months. No patients were lost to follow up, at the end of the follow-up, success was observed in 52 patients, 10 presented with recurrence after LIFT. In all failure cases, the median time interval to recurrence was three months (1-12). All recurrent fistulas became intersphincteric fistulas. Among the cases with failure, eight male patients were cured by single fistulotomy approach, and two female were cured by cutting seton.

**TABLE 1:** Patient›s information and fistula characteristics (n=62)

Patient and fistula characteristics	n	percentage
Median age (range)	34(22-63)	
Gender		
Male	43	69.4
Female	19	30.6
Previous history of operation		
Incision and drainage of anal abscess	8	12.9
Thread-drawing of anal abscess	10	16.1
Smoking status		
Current smoker	17	27.4
Current non-smoker	45	72.6
Types of complex fistula		
High transsphincteric fistula	41	66.1
High Intrasphincter fistula	4	6.5
Anterior anal fistula in female		
Low transsphincteric fistula	11	17.7
Intrasphincter fistula	6	9.7
Location of fistula		
Anterior	22	35.5
Posterior	11	17.7
Lateral	19	30.6
Horseshoe fistula	8	12.9
Success		
Success	52	83.9
Failure	10	16.1

 The changes of anorectal pressure three months before and after operation were not obvious; neither were the anal resting pressure and maximum anal contractive pressure shown in Table 2. All the patients received Cleveland Clinic Florida Fecal Incontinence (CCF-FI) evaluation. The results showed that the autonomous control of anal sphincter of 62 cases were normal (CCF-FI score: 0).

**TABLE 2:** Comparison of anorectal pressure of patients with modified LIFT surgery before and after the operation (c±S)

Anorectal pressure	Before the operation	After the operation	t	p
Anal resting pressure(mmhg)	55.61±9.53	55.37±9.56	0.786	0.079
Anal contractive pressure(mmhg)	122.08±19.03	121.77±16.92	0.701	0.486

## DISCUSSION

A total of 62 patients underwent modified LIFT surgery for complex fistula-in-ano and were followed up for more than one year. No complex fistula-in-ano was found at the follow-up ended, 10 cases became intrasphincter fistula. The total cure rate was better than the existing published results of the complex fistula-in-ano treated with LIFT surgery. Possible causes of the formation of intersphincteric fistula are: 1) infections caused by other diseases round perianal region; 2) inadequate drainage due to accumulated blood and effusion; 3) residual necrosis and infected tissues in the intersphincteric groove; 4) intraoperative injury of internal anal sphincter and anal canal mucosa; 5) incomplete ligation of the internal sphincter fistula or necrosis of the residuals resulting in intersphicteric infection. Tan *et al.* ^16^ said that the incision of LIFT surgery located interior to the anal verge was small and deep, which could accumulate blood or effusion and increase postoperative incision infection and dehiscence. Van onkelen *et al.* ^17^ suggested that it might be the result of persistent intersphincteric infection caused by incomplete ligation of fistula at the side of internal anal sphincter during the operation. Wallin *et al.* ^18^ believed the identification of intersphincteric fistula and the complete ligation of fistula were the difficulties of LIFT surgery and the main reasons for operation failure (postoperative persistent infection of intersphincteric incision). Mohanlal Khadia *et al.* ^9^ thought possible to induce a failed ligation if the fistula was rather thin, deep or thick. In a conventional LIFT surgery for fistula ligation, because of the inconsistent thickness and fibrosis of intersphincteric fistulas, simple ligation often fails to completely tighten the fistula. The ligature then ruptures or falls off, thus the operation falls flat. Taking these complex situations into consideration, we dissected the anal skin and incised deeply into the intersphincteric groove to keep it away from the medial side of anal verge which is easy to cause concurrent infection. This measure reduced the incidence of incision infection and dehiscence purse-string suture for fistula ligation prevented many complications caused by ligature rupture and incomplete ligation due to insufficient fibrosis, overly thin fistula or ligature’s falling off.

Bastawrous A *et al.* ^1^ improved LIFT surgery to prevent infection of sphincter incision and fistula formation between sphincters. In their surgery, fistula tract was ligated at external sphincter, and internal sphincterotomy was performed along fistula tract. Their cure rate was 71.42%, close to 76.19% of ours. Compared with conventional LIFT surgery, they removed part of the internal sphincter. So, a long-term follow-up should be studied to clarify the effect on the removed internal sphincter on anal function.

Although there was not any completely failed case in our study, reasons for complete failure include: 1) incomplete ligation along external sphincter cannot effectively close the fistula, and the infected fistula may develop from intersphincteric space to outside sphincter; 2) infection of residual fistulas appear on the lateral border of external sphincter^15^. Liu *et al.* ^11^ found the length of fistula was inversely proportional to the cure rate of LIFT surgery. The fistula less than 3 cm was considered as a risk factor for surgery failure. The longer the fistula was, the higher the possibilities of persistent residual epithelialization and infection of necrotic tissue residues were, therefore the difficulty of this cure and the risk of recurrence increased. Curettage and drainage are major solution of residual fistulas after LIFT surgery^10^. However, studies have showed that simple curettage neither completely removes the existing epithelialization tissues, nor maintains the unobstructed drainage of residual fistulas. As a result, fistula grows a non-healing communication^12^.

For the external sphincter fistula gap, Ellis *et al.* ^2^ designed BioLIFT surgery which added biological patch to LIFT; its cure rate reached up to 94%; Han *et al.* ^6^ combined LIFT with bio prosthetic anal fistula plug (LIFT + Plug) for anal fistula, showing 95% cure rate at early stage, with little gas leakage. Both biological patch and anal fistula plug filled the gap of the external sphincter fistula. These two surgeries showing higher cure rate probably indicate the trend in the treatment of complex anal fistula. But, it is a pity that the high cost of biological patch and anal fistula plug prevent them from being widely used in clinic now. Compared with conventional LIFT surgery, our modified procedure does not bring extra medical materials or treatment fee, and we did not find any completely failed case or recurrence. The external sphincter fistula gap is difficult to be completely closed, and the residual fistulas cannot be simply removed by curettage either. But, since they are the key to reduced recurrence of LIFT, we applied purse-string suture in the ligation to complete the external sphincter fistula gap the once. Not only did it close the fistula gap passing through the external sphincter, it also indirectly repaired the external sphincter defect. As for the residual fistulas between the external opening and the intersphincteric space, we removed it in a tunnel-based way. The fistula was completely withdrawn, and the surface of the distal wound was of radial shape with large mouth and small bottom. The distal fistula thus could be removed throughly, drainage would not be obstructed, and change of dressing would be more convinent. They together reduced the residual lesions and the failure rate of incision recovery caused by accumulated blood and effusion to the max. If it is a horseshoe anal fistula, curved incision will be made on the main tract identified by MRI scan or examined by finger. Purse-string suture in then performed to tie up the fistula, and branch in the external sphincter is tunneled. Besides, several radial incisions are made on the outer sphincter through which longer fistula pass. Afterwards, we tunnel the fistula to remove it and fully drain off the effusions. Among the cases we collected, there were eight patients with horseshoe anal fistula. Three of them developed postoperative sphincter fistula. The total success rate was 62.5%, superior to 40% of the horseshoe anal fistulas reported^13^. We believe the reason for our better result is the tunneled removal of the fistula, which reduces the recurrence induced by the residual fistula after conventional scraping and thread-drawing therapies. But, we still need to investigate the technique that can improve the success rate of LIFT surgery for horseshoe anal fistula in the following study.

We cannot deny that there are some limitations in present study. As a retrospective analysis, there is significant selection bias. The complex fistula-in-ano cases collected in the study have not included all the types, like suprasphincteric and extrasphincteric fistulas, and recurrent fistula is not included in the study either, for the injuries of the sphincter in the last operation.

Multi-centered randomized controlled studies are needed to make more accurate evaluation on the effectiveness and safety of the modified LIFT surgery.

## CONCLUSION

Our modified LIFT surgery for complex fistula-in-ano effectively reduces the failure and recurrence rate of LIFT and protect the function of anal sphincter and anus with acceptable long-term outcomes. 
